# Higher values of triglycerides:HDL-cholesterol ratio hallmark disease severity in children and adolescents with sickle cell anemia

**DOI:** 10.1590/1414-431X20198833

**Published:** 2019-10-14

**Authors:** R.S. Teixeira, M.B. Arriaga, R. Terse-Ramos, T.A. Ferreira, V.R. Machado, M.R. Rissatto-Lago, P.S. Silveira-Mattos, N. Boa-Sorte, A.M.T. Ladeia, B.B. Andrade

**Affiliations:** 1 Escola Bahiana de Medicina e Saúde Pública, Salvador, BA, Brasil; 2 Departamento de Pediatria, Faculdade de Medicina, Universidade Federal da Bahia, Salvador, BA, Brasil; 3 Instituto Gonçalo Moniz, Fundação Oswaldo Cruz, Salvador, BA, Brasil; 4 Multinational Organization Network Sponsoring Translational and Epidemiological Research (MONSTER) Initiative, Fundação José Silveira, Salvador, BA, Brasil; 5 Departamento de Ciências da Vida, Universidade Estadual da Bahia, Salvador, BA, Brasil; 6 Universidade Salvador, Laureate International Universities, Salvador, BA, Brasil

**Keywords:** Sickle cell disease, Lipoproteins, Cholesterol, Triglycerides, Hydroxyurea, Endothelial function

## Abstract

Dyslipidemia has been described in sickle cell anemia (SCA) but its association with increased disease severity is unknown. Here, we examined 55 children and adolescents with SCA as well as 41 healthy controls to test the association between the lipid profiles in peripheral blood and markers of hemolysis, inflammation, endothelial function, and SCA-related clinical outcomes. SCA patients exhibited lower levels of total cholesterol (P<0.001), low-density lipoprotein cholesterol (LDL-c) (P<0.001), and high-density lipoprotein cholesterol (HDL-c) (P<0.001), while displaying higher triglyceride (TG) levels and TG/HDL-c ratio values (P<0.001). TG/HDL-c values were positively correlated with lactate dehydrogenase (P=0.047), leukocyte count (P=0.006), and blood flow velocity in the right (P=0.02) and left (P=0.05) cerebral artery, while being negatively correlated with hemoglobin levels (P<0.04). Acute chest syndrome (ACS) and vaso-occlusive events (VOE) were more frequent in SCA patients exhibiting higher TG/HDL-c values (odds ratio: 3.77, P=0.027). Multivariate logistic regression analysis confirmed independent associations between elevated TG/HDL-c values and SCA. Thus, children and adolescents with SCA exhibited a lipid profile associated with hemolysis and inflammatory parameters, with increased risk of ACS and VOE. TG/HDL-c is a potential biomarker of severity of disease.

## Introduction

Sickle cell anemia (SCA) is a hemoglobinopathy of autosomal recessive inheritance that manifests with hemolysis, vaso-occlusive crises, progressive organic damage, and early death (1). SCA pathophysiology is complex and involves activation of leukocytes and intricate interactions between abnormal erythrocytes and the vascular endothelium (2,3). In SCA, the dyslipidemia profile characterized by lower levels of total cholesterol, low-density lipoprotein cholesterol (LDL-c), high-density lipoprotein cholesterol (HDL-c), and high levels of triglycerides (TG) has been described, but the impact of these changes in the clinical picture needs to be better understood (4). In some clinical settings, serum cholesterol is an important parameter for assessment of disease severity and/or progression, with lower values usually being indicative of increased risk of death (5). Previous studies in adult patients with SCA have described a positive correlation between levels of TG and circulating concentrations of markers of hemolysis and inflammation, whereas TG/HDL-c ratio values are associated with endothelial dysfunction (6). Of note, hypertriglyceridemia in this patient population is considered a risk factor for pulmonary hypertension (6), a leading cause of death in adults with SCA. However, a detailed role of the TG/HDL-c ratio and associations with the occurrence of vascular events has not been reported in pediatric populations with SCA.

In the present study, we characterized the lipid profile of children and adolescents with SCA and tested its association with markers of hemolysis, inflammation, endothelial dysfunction, and clinical aspects of the disease.

## Material and Methods

### Ethics statement

The study was approved by the Ethics Committee of the Escola Bahiana de Medicina e Saúde Pública (EBMSP), Salvador, Brazil (protocol number 568.913/2014). Written informed consent was obtained from each participant or legal guardian at study enrollment, according to the resolution 466 of the National Health Council (BRASIL, 2012). All institutions participating in the study authorized data collection. All clinical investigations were conducted according to the principles of the Declaration of Helsinki.

### Study design and sample selection

This study was comprised of secondary analyses of data collected and expanded on previously completed research (7), which included children and adolescents aged between 6 and 18 years, diagnosed with SCA, with or without the use of hydroxyurea and age-matched healthy children. The participants were assigned to two reference centers for the treatment of hematological diseases, including the Hematology Outpatient Clinic of the Magalhães Neto Ambulatory-HUPES Complex of the Federal University of Bahia Medical School, and Hematology and Hemotherapy Foundation of Bahia (HEMOBA). The healthy children and adolescents were registered in the general preventive pediatrics clinic of Roberto Santos General Hospital (HGRS)/Bahia and EBMSP or the adolescent clinic of the Magalhães Neto Outpatient Clinic-HUPES. These institutions are part of the Unified Health System (Sistema Único de Saúde, SUS), which provides publicly funded healthcare to the Brazilian population, mostly people with low economic status.

### Inclusion and exclusion criteria

Individuals with SCA aged between 6 and 18 years, with SCA diagnosed by Hb electrophoresis and/or high-performance liquid chromatography, without acute complications related to the disease or infectious conditions one month before inclusion, without chronic diseases, non-SCA (HbAA), and with BMI for age below +2 of the z-score according to the 2007 World Health Organization (WHO) charts (8) were enrolled in the study. Individuals with SCA were excluded if they had a cerebrovascular incident or blood transfusion 3 months before the study. The exclusion criteria for the control group included acute infectious conditions, dyslipidemia, and obesity.

The demographic and clinical parameters were evaluated through a standardized survey and medical records. The physical examinations included anthropometric measurements, vital signs, and peripheral oxygen saturation data.

### Event definitions

Vaso-occlusive episodes (VOE) were described as pain symptoms warranting analgesia (9). Acute chest syndrome (ACS) was defined as new pulmonary infiltrate involving at least one segment of the lung and isolated atelectasis with one or more associated respiratory symptoms (10,11).

### Laboratory data

Laboratory data were collected after the endothelial dysfunction test and after a fasting period of at least 8 h. The lipid profile included total cholesterol (TC), HDL-c, LDL-c, and triglycerides (TG) measured by enzymatic methods, and high sensitivity C-reactive protein (hs-CRP) using the turbidimetry method in a reference laboratory. The other examinations were part of the outpatient examination, including the transcranial Doppler. This test is performed annually in children with SCA from 2 years of age. A study by Adams et al. (12) defined values for blood flow velocity: up to 170 cm/s (normal); from 171 to 200 cm/s (conditional); and greater than 200 cm/s (critical/abnormal).

### Evaluation of endothelial function

According to our previously described technique to evaluate endothelial function (7), a protocol established under the guidelines for ultrasonographic evaluation of the forearm (13) was used. The examinations were performed using a VIVID 3 ultrasound scanner (General Eletric Company, Israel) with a 12 MHz multi-frequency transducer. The endothelium-dependent vasomotor function was assessed using flow-mediated vasodilation and measured using reactive hyperemia.

The examinations were performed by a specially trained physician with proven experience in the technique (14). Throughout the examination, a synchronized electrocardiogram was also obtained.

Endothelial dysfunction was defined as a flow-mediated vasodilation value below the 10th percentile of the healthy group, as described by Jarvisalo et al. (15) and Andrade et al. (16). The dyslipidemia criteria were defined according to the V Brazilian Directive on Dyslipidemia and Prevention of Atherosclerosis (17,18)

### Hydroxyurea (HU) treatment of SCA patients

For the use of HU in patients with SCA, the recommendations of the treatment protocol of the Ministry of Health of Brazil were followed, which consisted of an initial dose of 15 mg·kg^−1^·day^−1^ and a maximum tolerated dose of 35 mg·kg^−1^·day^−1^. The mean dose of HU was 20 mg·kg^−1^·day^−1^.

### Statistical analysis

Mean and standard deviation were used to characterize the dependent and independent variables. Student's *t*-test, Spearman correlations, and chi-squared test were used to compare independent sample means, associations, and proportions, respectively. Receiver operator characteristics (ROC) curves were employed to test the accuracy of TG/HDL-c ratio values to distinguish SCA patients presenting with ACS and/or VOE history from those who did not. Finally, a logistic regression was performed to evaluate the independent associations between clinical and laboratory variables and the presence of SCA. All analyses were pre-specified. Comparisons displaying P values <0.05 were considered statistically significant. The data analysis was performed using IBM SPSS Statistics for Windows, version 23.0 (IBM Corp., USA).

## Results

### Clinical characteristics of study participants

This study included 55 patients with SCA (HbSS) and 41 healthy children and adolescents (HbAA; control group). In the SCA group, 24 (43.6%) subjects reported use of HU. SCA patients were similar to healthy individuals with regard to age. Frequency of male individuals was higher in the group of SCA. In addition, both absolute and z-score-normalized body mass index (BMI) values were lower in the SCA patients compared to those in the control group (Table 1).

**Table 1.** Clinical characteristics of the study participants.

Characteristics	SCA patients (n=55)	Controls (n=41)	P value
Age (years)	12.44±3.2	11.41±3.17	0.123
Males (n, %)	31 (56.36)	14 (34.14)	0.039
BMI (kg/m^2^)	16.74±2.3	18.61±3.96	0.011
Z score BMI (AU)	-0.93±1.0	-0.12±1.36	0.003

Data are reported as means±SD or number (%). The *t*-test or chi-squared test were used to compare groups. SCA: sickle cell anemia; BMI: body mass index; AU: arbitrary units.

### Hematological assessment of SCA

We next compared the study groups with regard to a number of laboratory parameters. As expected, hematological evaluation revealed that patients with SCA exhibited on average lower levels of hemoglobin compared to healthy individuals. Mean corpuscular volume values were also significantly higher in SCA patients. Reticulocyte counts were elevated in SCA compared to controls. SCA was associated with increased platelet and leukocyte counts (Table 2).

**Table 2.** Hematological characteristics of the study participants.

Parameter	SCA patients (n=55)	Controls (n=41)	P value
RBC (× 10^6^/µL)	2.69±0.49	4.64±0.36	<0.001
Hemoglobin (g/dL)	8.04±0.84	13.13±1.1	<0.001
Hematocrit (%)	23.94±3.09	39.36±3.18	<0.001
Mean cell volume (fL)	90.81±10.83	83.42±6.78	0.007
Mean cell hemoglobin concentration (pg)	33.59±4.18	33.14±1.34	0.503
Reticulocyte count (%)	7.63±4.89	0.8±0.23	<0.001
Leukocyte count (× 10^9^/L)	12.15±37.11	72.13±15.33	<0.001
Neutrophil count (%)	48.82±16.32	50.47±13.08	0.706
Monocyte count (%)	8.15±3.34	7.75±2.13	0.564
Platelet count (× 10^9^/L)	454.70±139.00	281.17±47.32	<0.001

Data are reported as means±SD. Chi-squared test was used to compare groups. SCA: sickle cell anemia; RBC: red blood cells.

### Biochemical assessment of SCA

SCA patients displayed increased levels of serum lactate dehydrogenase (LDH) compared to healthy controls. While examining biomarkers of hepatocyte stress, we observed that SCA was associated with substantially higher levels of alanine aminotransferase (ALT) and aspartate transaminase (AST). Total bilirubin as well as indirect bilirubin values were more elevated in SCA patients (Table 3).

**Table 3.** Biochemical characteristics of the study participants.

Parameter	SCA patients (n=55)	Controls (n=41)	P value
Aspartate aminotransferase (U/L)	50.91±21.93	23.16±12.28	<0.001
Total bilirubin (mg/dL)	3.26±1.90	0.43±0.26	<0.001
Direct bilirubin (mg/dL)	0.7±0.75	0.1±0.08	0.012
Indirect bilirubin (mg/dL)	2.63±1.87	0.33±0.19	<0.001
Lactate dehydrogenase (U/L)	1184.47±576.68	387.3±32.77	<0.001
Alanine aminotransferase (U/L)	27.05±17.19	16.79±8.79	0.003
C-reactive protein (mg/dL)	3.79±4.27	2.14±4.08	0.049

Data are reported as means±SD. The *t*-test was used to compare groups. SCA: sickle cell anemia.

Assessment of the lipid profile revealed that SCA patients exhibited increased circulating levels of TG. Furthermore, SCA was associated with decreased values of total cholesterol, LDL-c, and HDL-c. The TG/HDL-c ratio has been used as a marker for incidence and extent of coronary artery disease in both men and women (16). In the present study, SCA patients exhibited higher values of TG/HDL-c ratio than healthy controls (Table 4).

**Table 4.** Lipid profile of the study participants.

Parameter	SCA patients (n=55)	Controls (n=41)	P value
Total cholesterol (mg/dL)	119.16±23.66	154.99±27.33	<0.001
HDL-c (mg/dL)	33.44±14.25	47.23±11.63	<0.001
LDL-c (mg/dL)	67.5±22.02	90.43±22.52	<0.001
Triglycerides (mg/dL)	105.57±43.16	74.07±25.87	<0.001
Triglycerides/HDL-c (AU)	3.64±2.15	1.7±0.83	<0.001

Data are reported as means±SD. SCA: sickle cell anemia; HDL-c: high-density lipoprotein cholesterol; LDL-c: low-density lipoprotein cholesterol; AU: arbitrary units. The *t*-test was used to compare groups.

In SCA patients, hemoglobin levels were inversely correlated with values of TG/HDL-c ratios (r=−0.389, P=0.04) and positively correlated with LDH (r=0.30 P=0.047). Interestingly, we observed a positive correlation between TG/HDL-c values and total leukocyte counts (Figure 1). TG/HDL-c values were also positively correlated with concentrations of values of blood flow velocity in the right (r=0.376, P=0.02) and left (r=0.296, P=0.05) cerebral arteries, examined by transcranial Doppler. These findings suggested that the lipid profile in SCA likely reflected the degree of systemic inflammation and potentially impacted clinical presentation.

**Figure 1.** Spearman correlations analysis of severity parameters and triglycerides (TG):high-density lipoprotein cholesterol (HDL-c) ratio in sickle cell anemia (SCA) patients. MCA: middle cerebral artery.

### Assessment of endothelial dysfunction and inflammation in SCA

SCA patients presented with higher values of CRP, indicating augmented systemic inflammation (Table 3). Flow-mediated vasodilation values were on average lower in the SCA patients compared to controls (10.9%±5.9 *vs* 15.8%±8.3, P=0.002), indicating a lower endothelium-dependent vasodilator capacity.

### Assessment of the flow velocity in the middle cerebral artery in SCA

The flow velocity in the right middle cerebral artery was 130 cm/s (IQR: 112–148 cm/s) and the flow velocity in left middle cerebral artery was 131 (109–156) cm/s assessed by transcranial Doppler. The transcranial Doppler ranking was normal in 56.4% (n=31), conditional in 10.9% (n=6), not normal in 5.5% (n=3), and asymmetric in 3.6% (n=2).

### Clinical events in SCA

VOE occurred in 92.7% (51) of SCA patients, with 42 individuals demanding emergency care (76.4%) and 35 (63.6%) VOE requiring hospitalization. ACS occurred in 35 (67.3%) patients.

Univariate analyses indicated that clinical, hematological, and lipid parameters were associated with SCA (Tables 1, 2, and 4). Multivariate regression analysis confirmed that male sex and TG/HDL-c are independently associated with increased odds for SCA (Figure 2).

**Figure 2.** Variables associated with sickle cell anemia (SCA). Multivariate regression model of variables shown in Tables 1, 4, and 5 that displayed univariate P value ≤0.2.

We used receiver operator characteristics (ROC) curve analysis to test if TG/HDL-c could be used as a marker of SCA clinical severity. We found that a TG-HDL-c value below 2.93 had a sensitivity of 78% and a specificity of 71% for identifying SCA patients who had presented ACS and/or VOE from those who did not (Figure 3). Patients with SCA and TG/HDL-c ratio above the cut-off value 2.93 presented higher numbers of ACS events (n=24 (70.6%) *vs* n=10 (29.4%), P=0.027), OR=3.77, 95%CI: 1.135–12.53 and more VOE (n=32 (62.7%) *vs* n=18 (35.3%), P= 0.057).

**Figure 3.** Using triglycerides (TG):high-density lipoprotein cholesterol (HDL-c) ratio values in sickle cell anemia (SCA) patients to identify individuals with acute chest syndrome (ACS) and/or vaso-occlusive episodes (VOE). **A**, TG/HDL-c values were compared between the ACS+VOE group and controls using the Mann-Whitney *U* test. Lines represent median values and interquartile ranges. **B**, Receiver operator characteristics (ROC) curve analysis was employed to test the accuracy of TG/HDL-c values to discriminate between individuals with ACS+VOE history and controls. **C**, Detailed information obtained from the ROC curve, such as area under curves (AUC), P value of the ROC curves, cut-off value, and sensitivity and specificity with the 95% confidence interval (CI).

### Impact of HU treatment on SCA

In the group of SCA patients treated with HU, 75% (n=18) used this drug for less than 3 years, 58.3% (n=14) for less than 2 years, and 8.3% (n=2) for less than six months. Treatment with HU in SCA patients did not substantially affect levels of total cholesterol, HDL-c, LDL-c, TG, and TG/HDL-c ratio (Table 5).

**Table 5.** Characteristics of sickle cell anemia (SCA) patients stratified by hydroxyurea (HU) treatment status.

Parameter	SCA non-HU (n=30)	SCA + HU (n=24)	P value
Hemoglobin (g/dL)	7.9±0.8	8.2±0.9	0.29
Fetal hemoglobin (g/dL)	6.7±5	8.6±6.4	0.39
Mean cell volume (fL)	86.7±9.8	94.9 ±10.9	0.01
Leukocyte count (× 10^9^/L)	12.6±3.2	11.7±4.3	0.41
Platelet count (× 10^9^/L)	458±106	469±148	0.75
Reticulocyte count (%)	8±5	7.4±5	0.70
Neutrophils (%)	46.5±4	50.8±3	0.40
Lactate dehydrogenase (U/L)	1369±636	980±432	0.03
Aspartate aminotransferase (U/L)	55±21	46±22	0.20
Alanine aminotransferase (U/L)	27.9±18.5	26.1±16	0.72
C-reactive protein (mg/dL)	4.64±5.10	3.20±3.46	0.25
Total cholesterol (mg/dL)	124±22	115±26	0.88
LDL-c (mg/dL)	67±24	69.6±23	0.50
HDL-c (mg/dL)	34.6±9.4	33±5.7	0.70
Triglycerides (mg/dL)	104±47	99.5±28.6	0.40
Triglycerides/HDL-c ratio (AU)	3.95±2.3	3.2±1.9	0.22
Flow mediated dilatation (%)	11.6±5.7	10±5.7	0.32

Data are reported as means±SD. HU: hydroxyurea; HDL-c: high-density lipoprotein cholesterol; LDL-c: low-density lipoprotein cholesterol. The *t*-test was used to compare groups.

There was a significant difference in the mean globular volume between the SCA non-HU groups and SCA+HU by increasing hydration of the erythrocyte, produced by the use of HU and a significant difference in the lactic dehydrogenase levels by reduction of hemolysis. There was a slight increase, although not statistically significant, in fetal hemoglobin. Platelet, leukocyte, and neutrophil counts (Table 5) were also not altered in the group of individuals taking HU.

## Discussion

Assessment of lipid profile in SCA and its relationships with hemolysis, endothelial dysfunction, and systemic inflammation can provide insights on the risk for vascular damage and clinical severity (19). In the present study, we found lower levels of total cholesterol, HDL-c, and LDL-c in SCA patients. In contrast, higher levels of triglycerides were observed in SCA, consistent with the findings of previous studies that included adults and children with SCA (20 [Bibr B21]–22).

Cholesterol plays an important role in cellular metabolism, including cell membrane synthesis; membranes are comprised of 52% proteins, 40% phospholipids and cholesterol, and 8% carbohydrates (23). Low plasma levels of cholesterol have been reported in several types of acquired and hereditary hematological disorders, including megaloblastic anemia, iron deficiency anemia, aplastic anemia, anemia associated with liver disease, hereditary spherocytosis, SCA, and thalassemia (4). The main mechanisms underlying this phenomenon are the consumption of cholesterol for red blood cell synthesis and serum cholesterol dilution due to the decrease in erythrocyte mass with increased plasma content. Belcher et al. (19) demonstrated that sickle-cell LDL was more susceptible to oxidation than control LDL and that LDL-vitamin E levels were significantly lower in SCA patients compared with control subjects. In addition, the cytotoxicity of partially oxidized LDL to endothelial cells suggests that oxidized LDL may be a marker of vasculopathy and oxidative stress (19).

In this study, the association between the lipid markers and inflammation were demonstrated as a negative correlation between cholesterol and hs-CRP and a positive correlation between TG/HDL-c and leukocytes. In SCA, hs‐CRP has been described as a low‐grade marker of inflammation, correlated to episodes of VOE (24). Leukocyte count is also known as an independent factor associated with SCA clinical severity. Patients with elevated leukocyte counts are more likely to die at a young age (25) and are more susceptible to develop ACS (29) and silent cerebral infarction (26).

TG/HDL-c values were positively correlated with LDH levels and negatively correlated with hemoglobin concentrations in the study reported here. Hemolysis compromises the nitric oxide availability and is considered one of the main mechanisms of vasculopathy and chronic complications such as pulmonary hypertension, priapism, stroke, and leg ulcers (27). There was a significant positive correlation between TG/HDL-c ratio and blood flow velocity in the right and left cerebral arteries by transcranial Doppler. Blood flow velocity measured by transcranial Doppler is an important predictor of stroke risk, which increases with increasing maximum flow velocity (28). Stroke is one of the main causes of morbidity and mortality in SCA, affecting mainly children, especially those under 10 years of age.

ACS predominated in the SCA group with very high TG/HDL-c ratio values. This finding is in agreement with a previous study that reported this marker to be associated with risk for other diseases (18,29). ACS is the second cause of hospitalization in patients over 2 years of age, the main cause of hospitalization in intensive care units, and the main cause of mortality in SCA (25,30). In this study, SCA patients were 10 times more likely than healthy controls to have elevated TG/HDL-C ratios. These data reinforce the pathophysiological interrelationships between hemolysis, inflammation, and lipoproteins in SCA, and reinforce the idea of the potential role of the lipid profile, especially the TG/HDL-c, as a marker of vascular events in children and adolescents with SCA.

There was no difference in the lipid profile between SCA patients with or without HU treatment. Taking into account that HU decreases hemolysis and perhaps inflammation, these mechanisms would decrease cholesterol consumption and oxidation, respectively, producing an impact of the hypocholesterolemia observed in SCA (6). The similarities between the groups of individuals treated or not with HU in leukocyte, platelet, and neutrophil counts and the non-significant elevation of fetal hemoglobin in the HU group suggest that HU treatment was suboptimal with patients being undertreated. Adherence was not evaluated herein and there is a possibility of treatment interruptions due to the lack of availability of medications in the public health system. The study design did not allow us to definitively conclude whether HU treatment interferes with lipid levels in SCA, as we did not measure blood lipids before drug administration.

In summary, our findings demonstrated that children and adolescents with SCA in a stable disease state presented changes in lipid metabolism characterized by low levels of total cholesterol, LDL-c, and HDL-c as well as high TG levels and TG/HDL-c ratio. The correlations between the levels of lipoproteins and markers of hemolysis and inflammation suggested the involvement of these mechanisms in the dyslipidemia profile of patients with SCA (27). The high frequency of ACS and VOE in SCA patients exhibiting elevated TG/HDL-c ratio values highlights an association between dyslipidemia and vascular events. Lastly, associations between the TG/HDL-c values and leukocyte counts, LDH concentrations, hemoglobin levels, blood flow velocity values in the middle cerebral artery, and ACS, reinforce the potential of the TG/HDL-c ratio as an early marker of clinical severity and may be implemented as a point-of-care assessment approach.
